The article "Eupafolin induces apoptosis and autophagy of breast cancer cells through PI3K/AKT, MAPKs and NF-κB signaling pathways" was retracted in 2021. Reason: duplicated images.

# Eupafolin induces apoptosis and autophagy of breast cancer cells through PI3K/AKT, MAPKs and NF-κB signaling pathways

**DOI:** 10.1038/s41598-021-00945-9

**Published:** 2021-11-02

**Authors:** Jiahui Wei, Yu Ding, Xinmiao Liu, Qing Liu, Yiran Lu, Song He, Bao Yuan, Jiabao Zhang

**Affiliations:** 1 Department of Laboratory Animals, College of Animal Sciences, Jilin University, Changchun, 130062 Jilin People’s Republic of China; 2 The Second Clinical School of Medicine, Guangdong Provincial Hospital of Chinese Medicine, Guangdong Provincial Hospital of Chinese Medicine-Zhuhai Hospital, Guangzhou University of Chinese Medicine, Guangzhou, 510120 Guangdong China

**Keywords:** Cancer, Cell biology, Drug discovery, Molecular biology, Zoology, Oncology

## Abstract

Eupafolin is a flavonoid that can be extracted from common sage. Previous studies have reported that Eupafolin has antioxidant, anti-inflammatory and anti-tumor properties. However, no studies have investigated the role of Eupafolin in breast cancer. Herein, we investigated the effect of Eupafolin on two human breast cancer cell lines, as well as its potential mechanism of action. Next, the data showed that proliferation, migration and invasion ability of breast cancer cells that were treated with Eupafolin was significantly reduced, while the apoptosis rate was significantly increased. In addition, Eupafolin treatment caused breast cancer cell proliferation to be blocked in the S phase. Moreover, Eupafolin significantly induced autophagy in breast cancer cells, with an increase in the expression of LC3B-II. PI3K/AKT, MAPKs and NF-κB pathways were significantly inhibited by Eupafolin treatment. Additionally, 3-MA (a blocker of autophagosome formation) significantly reduced Eupafolin-induced activation of LC3B-II in breast cancer cells. Furthermore, Eupafolin displayed good in vitro anti-angiogenic activity. Additionally, anti-breast cancer activity of Eupafolin was found to be partially mediated by Cav-1. Moreover, Eupafolin treatment significantly weakened carcinogenesis of MCF-7 cells in nude mice. Therefore, this data provides novel directions on the use of Eupafolin for treatment of breast cancer.

## Introduction

Breast cancer is one of the most dangerous invasive cancers among women, with a high prevalence worldwide^1^. Improving the ability to treat breast cancer requires ongoing clinical and basic research. The recurrence rate of breast cancer is very high, and many patients develop drug resistance, which leads to side effects^2^. Therefore, identifying non-toxic and efficacious natural compounds for the treatment of breast cancer is of utmost importance.

Chinese medicine has been widely used in China. Due to the non-toxic effects and efficacy of Chinese medicine, it is often used in combination with other, western medicines. Eupafolin is a flavonoid that has anti-inflammatory, anti-viral, anti-angiogenesis and anti-tumor activities^3^. Previous studies have demonstrated that angiogenesis is important to the development of solid tumors. Therefore, anti-angiogenesis strategies can help develop novel treatment methods for solid tumors^4^.

Autophagy is an evolutionarily conserved lysosomal degradation pathway, and thus, normal levels of autophagy are needed for maintenance of cellular metabolism. However, autophagy can play a role in suppressing tumors as well as tumorigenesis, particularly under the conditions of nutrient or growth factor deficiency or hypoxia^5,6^. Previous studies have shown that inhibition of autophagy in tumor cells is further developed^7–9^. Beclin-1 and LC3 are commonly-used markers of autophagy. Herein, research on autophagy may be of great significance in the treatment of breast cancer.

Proteins that are involved in the PI3K/Akt pathway are abnormally expressed among several cancers, and have been directly associated with progression of breast cancer, gastric cancer, and pancreatic cancer, among others. The PI3K, NF-κB and MAPKs pathways are closely related to tumor proliferation and autophagy^10^. Several studies have shown that targeting this pathway through the use of drugs or drug combinations is effective in the treatment of tumors^11^. Thus, research on drugs that target PI3K/AKT, MAPKs and NF-κB pathway may be of great significance in the short and long-term management of breast cancer.

Therefore, we set out to identify the possible underlying mechanism of action of Eupafolin in breast cancer. Experimental results demonstrated that Eupafolin significantly inhibited the growth of breast cancer by the PI3K/AKT, MAPKs and NF-κB pathways, causing S-phase arrest, inhibiting angiogenesis and promoting apoptosis, which was partially mediated by Cav-1.

## Materials and methods

### Cell culture

MDA-MB-231, MCF-7 and human umbilical vein endothelial cells (HUVECs) were purchased from the Wuhan Punuosai Life Technology Co., Ltd. (Wuhan, China) and Shanghai Suran Biological Technology Co., Ltd. (Shanghai, China). All cells were grown in Dulbecco’s Modified Eagle’s Medium (DMEM), and high glucose was supplemented with 10% fetal bovine serum (FBS, Gibco) in a humidified atmosphere of 5% CO_2_ at 37 °C. Eupafolin (purity ≥ 99%) was purchased from Yuanye Biotechnology. In this study, Eupafolin was dissolved in dimethyl sulfoxide (DMSO, Beijing Solarbio Science & Technology Co., Ltd) at different concentrations (0, 25, 50 and 100 μM). Subsequently, cells were treated with Eupafolin for different time periods. The siRNA-Cav-1 (Suzhou Jima) was transfected into breast cancer cells using Lipofectamine 2000™ reagent (Suzhou Jima). Rapamycin (RA) and 3-methyladenine (3-MA) were purchased from (MCE).

### Cell counting kit-8 and colony formation assay

In brief, 5000 cells were seeded onto 96-well plates, treated with 0, 25, 50 and 100 µM Eupafolin, and then incubated for 24, 48 and 72 h. Then, a microplate reader was utilized to measure the absorbance at 450 nm (TECAN). Then, cells with an adhesion rate > 90% (in logarithmic growth phase) were trypsinized, centrifuged, and resuspended for counting cells. Then, the cells were placed into 6-well plates at a density of 1,000 cells/well, and then placed into a 37 °C CO_2_ incubator for culturing. After 7 days of incubation, once the colonies were visible to the naked eye, they were removed from the 6-well plate, the culture medium was discarded, and 2 mL of methanol was added to each well for 30 min. Next, the methanol was discarded, and 1 ml of 0.1% crystal violet was added to each well for staining for three minutes. Finally, the purple crystals were washed away, and photos were taken with a digital camera. The colonies were counted under a light microscope.

### Transwell experiments

After Eupafolin treatment, cells were digested, resuspended in a serum-free medium, and adjusted to a density of 1 × 10^5^ cells/ml. Next, the transwells were placed in an incubator for 24 h. After that, the cells were removed and the medium was aspirated. In a new 24-well plate, 600 µl of 4% paraformaldehyde was added. The transwell was placed at 37 °C and cells were fixed for 30 min. The fixative solution was then removed and cells were stained at 37 °C using 0.2% crystal violet for 10 min. Then, the excess crystal violet was removed prior to microscopy. After the cells were dried, They were observed and counted under an inverted light microscope using a digital camera (magnification, ×80). The cell invasion test procedure was then used similarly to a cell migration assay.

### Cell cycle and apoptosis analysis

Apoptosis was quantified using the Annexin-V/FITC apoptosis detection kit, according to the manufacturer’s instructions (Ebisson). After drug treatment for 24 h, 2 × 10^6^ cells breast cancer cells and HUVECs were typsinized and then centrifuged at 800×*g* for five min. Then, the supernatant was discarded, resuspended in 300 µl 1× binding buffer, and a 5 µl sample was mixed with FITC-Annexin V. Then, 5 µl PI staining solution was added onto 200 µl 1× binding buffer five min prior to detection. Flow cytometry was conducted using FACS (Thermo Fisher Scientific, Inc). In the scatterplots, normal live cells (annexin-V-negative and PI-negative) were shown in the lower left quadrant, early apoptotic cells (annexin-V-positive and PI-negative) were shown in the lower right quadrant, and late apoptotic cells (annexin-V-positive and PI-positive) were shown in the upper right quadrant. The total apoptosis rate was calculated as the sum of the early and late apoptosis rates. For cell cycle analysis, after detaching the cells with trypsin, 2 × 10^6^ cells were added per cytometer tube and fixed in 70% ethanol at 4 °C overnight. Next, cells were resuspended in 500 µl 1× PI solution (Baihao) for 30 min at 37 °C. The analysis was then performed through the use of FACS (Thermo Fisher Scientific, Inc.). Finally, the results were assessed using ModFit LT (version 5.0; Verity Software House, Inc.).

### Reverse transcription-quantitative PCR (RT-qPCR).

According to instructions provided with the kit, the TRIzol reagent (Ruan) was utilized to extract total cellular RNA, and cDNA was generated through the use of Fastking RT kit (Tian gen Biotech Co., Ltd) with 2 µg of RNA. The primers used were designed using National Center for Biotechnology Information (NCBI). A RT-qPCR detection system (Eppendorf) was used to perform the RT-qPCR reactions using SYBR Green (Tian gen Biotech Co., Ltd.) and a total of 20 µl of reaction mixture. The 2^−ΔΔ^Cq method^12^ was utilized to assess gene expression.

### Angiogenesis analysis

The HUVECs were seeded onto a six-well plate. After 12 h, they were treated with Eupafolin at concentrations of 50 µM and 100 µM for 24 h. Then, we added matrigel to the 96-well plate (40 ml/well) and maintained it for 60 min. The cells were then digested with trypsin and diluted to 2 × 10^5^ cells/ml. Then, 100 µl of the cell suspension was added into each well of a 96-well plate. The cells were incubated at 37 °C for 6 h, and then visualized using randomly select several fields of view under an inverted microscope to observe the microtubule structure.

### Western blotting

After the cells were treated with Eupafolin for 24 h, they were harvested, and lysed on ice with RIPA lysis buffer for 30 min. Next, the BCA protein assay kit was utilized to determine the protein concentration. Furthermore, 5× loading buffer was added and the proteins were denatured at 95 °C for 10 min. Then, the protein sample was added to each well, separated using 10–12% SDS-PAGE at 120 V, and transferred to PVDF membranes. The membraned were probed with primary antibodies against Bcl-2 (cat. no. 4223), Bax (cat. no. 2772), cleaved caspase-3 (cat. no. 9661), PI3K (cat. no. 4257), p-PI3K (cat. no. 17366), Akt (cat. no. 4691), p-Akt (cat. no. 4060), LC3B (cat. no. 43566), Beclin-1 (cat. no. 3495), Caveolin-1 (cat. no.3267), CDK2 (cat. no.2546), CDK4 (cat. no.12790), Cyclin B1 (cat. no.4138) and GAPDH (cat. no. 5174) (all 1:1000, Cell Signaling Technology, Inc.) at 4 °C overnight. Subsequently, the membranes were washed three times with PBS, and then incubated with horseradish peroxidase (HRP)-conjugated secondary antibodies for 1 h at 37 °C. The protein bands were visualized using chemiluminescence assay kit (Dalian Meilun Biotechnology Co., Ltd.) and visualized with an imaging system (Tanon). All images were analysed as TIFF files with Image J k 1.45 for windows to build the figures. Graphs of signal intensity were obtained through band densitometry.

### RNA interference

Cav-1 siRNAs oligonucleotides were synthesized by Suzhou Gene Pharma Co., Ltd. (Suzhou, China). After breast cancer cells were seeded for 12 h, Cav-1 siRNA and lipo2000 were diluted with serum-free medium and added to the cells. The medium was changed to complete medium after 6 h, and the cells continued to culture in the 37 °C CO_2_ incubator.

### Experimental animal

All the experiments were approved by Animal Care and Use Committee of Jilin University (Grant No. SY202012006) and were carried out in compliance with the ARRIVE guidelines (http://www.nc3rs.org.uk/page.asp?id=1357). Overall, 10 female BALB/c nude mice (5 weeks old) were purchased from the Liaoning Changsheng Laboratory Animal Technology Co, Ltd. Then, 5 × 10^6^ MCF-7 cells in 100 ml PBS were subcutaneously inoculated into armpit of nude mice. Seven days after injection of cells, when the tumor had grown to approximately 50 mm^3^, mice were randomized into two groups (N = 5 in each group). The first group was treated with PBS, once daily, using an intraperitoneal injection. The second group was treated with 50 mg/kg Eupafolin, once daily with an intraperitoneal injection. Tumor size and weight are measured every 3 days. After 21 days post-inoculation, the nude mice were sacrificed and tissue was removed for further experiments.

### Statistical analysis

An unpaired Student’s t-test was utilized in the present study. The SPSS (v.20.0; IBM Corp.) software helped conduct statistical analysis. Data from three independent experiments were presented as the mean ± SD. Furthermore, a P-value of < 0.05 was considered statistically significant.

### Ethics approval

All experimental procedures were carried out in accordance with the Animal Care and Use Committee of Jilin University (Grant No. SY202012006).

### Consent to participate

All authors agree to participate.

## Results

### Eupafolin significantly inhibits breast cancer cell growth in vitro

First, we determined the inhibitory effect of Eupafolin on cell viability of breast cancer cells (MDA-MB-231, MCF-7). After treatment with Eupafolin for 24 h, 48 h and 72 h, the cell viability of breast cancer cells was detected using the CCK-8 method. The results demonstrated that, compared to the control group, the inhibitory effect of Eupafolin on cell viability of breast cancer cells was time and dose-dependent (Fig. 1A). Colony formation experiments were able to detect cell viability of tumor cells^13^. Results from the cell colony formation experiments showed that 50 μM and 100 μM Eupafolin was able to significantly inhibit colony formation after 10 days of treatment (Fig. 1B). In addition, results from the transwell experiments indicated that Eupafolin treatment significantly reduces the number of migration and invasion among the two types of cells (Fig. 1C). Contrastingly, mRNA expression of MMP2, MMP9, E-Cadherin and N-cadherin were significantly down-regulated after Eupafolin treatment (Fig. 1D). These results indicate that Eupafolin is able to significantly inhibit the viability of two breast cancer cell lines in vitro.

**Figure 1:** The effects of Eupafolin on the sensitivity of breast cancer cells. (**A**,**B**) MDA-MB-231 and MCF-7 cells were exposed to various concentrations of Eupafolin (0, 12.5, 25, 50 and 100 µM) for different times. The cell viability was determined using the Cell Counting Kit-8 assay and Colony formation assay. (**C**) MDA-MB-231 and MCF-7 cells were incubated with 50 or 100 μM of Eupafolin for 24 h, which was followed by transwell analysis for evaluation of migration and invasion. (**D**) RT-qPCR analysis of E-cadherin, N-cadherin, MMP2 and MMP9 in MDA-MB-231 and MCF-7 cells that were treated for 24 h with Eupafolin. Data are representative of three independent experiments, and are expressed as mean ± SD. P > 0.05 indicates non-significance; ***P < 0.001; **P < 0.01; *P < 0.05.

### Effects of Eupafolin on cell cycle phases, apoptosis and autophagy

In order to determine the effect of Eupafolin on cell cycle of breast cancer cells, we conducted flow cytometry. Results from flow cytometry demonstrated that Eupafolin significantly induces S phase arrest (32.84 to 48.13% for MDA-MB-231 and 24.72 to 32.30% for MCF-7) among breast cancer cells (Fig. 2A). Moreover, results demonstrate that mRNA and protein expression of CDK2, CDK4 and cyclin B1 were decreased in a dose-dependent manner after Eupafolin treatment (Fig. 2B,C). Moreover, Eupafolin treatment significantly increased the apoptotic ratio of breast cancer cells (Fig. 2D), and as the expression of cleaved caspase-3 and Bax increased, the expression of Bcl-2 decreased (Fig. 2E). Finally, Eupafolin treatment significantly increased the expression of LC3B-II and Beclin-1 in the two cells (Fig. 2F).

**Figure 2:** Effect of Eupafolin on the distribution of breast cancer cells in cell cycle phases, apoptosis and autophagy. MDA-MB-231 and MCF-7 cells were incubated with 50 or 100 μM of Eupafolin for 24 h. Next, all cells were collected for further analysis. (**A**) Flow cytometry analysis to determine the effect of Eupafolin on cell cycle arrest. (**B**,**C**) RT-qPCR and Western Blot analysis for CDK1, CDK2, CDK4 and Cyclin B1. Full-length images are presented in Supplementary Fig. 1. (**D**) Flow cytometry analysis for evaluation of apoptosis. (**E**) Western blot analysis of Bcl-2, cleaved caspase-3 and Bax. Full-length images are presented in Supplementary Fig. 2. (**F**) Western blot analysis of Beclin 1 and LC3-II. Full-length images are presented in Supplementary Fig. 3. Graphs of signal intensity were obtained through band densitometry and referred to GAPDH and control levels. Data are representative of three independent experiments and expressed as mean ± SD. P > 0.05 indicates non-significance; ***P < 0.001; **P < 0.01; *P < 0.05.

In order to further study the role of autophagy, we used Rapamycin (RA) and 3-methyladenine (3-MA)^14^. First, we tested the cell viability of Eupafolin-exposed human breast cancer cells after pre-treatment with 3-MA or RA. After RA pretreatment, the cell viability significantly decreased in comparison to Eupafolin treatment alone. Furthermore, 3-MA treatment was able to significantly reverse the inhibitory effect of Eupafolin on human breast cancer cell viability (Fig. 3A). Furthermore, results demonstrated that after 3-MA pretreatment, the induction of apoptosis, promoted by Eupafolin, could be reversed (Fig. 3B,C). Moreover, Western blot results showed that RA pretreatment significantly increases the expression of LC3B-II/I and Beclin-1 in breast cancer cells. Furthermore, 3-MA pretreatment reversed Eupafolin-induced increased expression of LC3B-II/I and Beclin-1 (Fig. 3D,E). Thus, Eupafolin-induced apoptosis could be changed by 3-MA and RA. Compared to the control group, Eupafolin pretreatment significantly reduced protein expression of p-PI3K, p-AKT, p-P38, p-ERK1/2 and p-NF-κB (Fig. 4A,B).

**Figure 3:** Eupafolin-induced apoptosis is accelerated by RA and inhibited by 3-MA in breast cancer cells. MDA-MB-231and MCF-7 cells were pre-treated with or without 3-MA (5 mM) or RA (5 μM) for 2 h, followed by treatment with Eupafolin for another 24 h. All cells were then harvested for further analyses. (**A**) CCK-8 analysis for cell viability calculation. (**B**,**C**) Flow cytometry analysis for apoptosis. (**D**,**E**) Western blot analysis for Beclin-1 and LC3-II/LC3-I expression. Full-length images are presented in Supplementary Fig. 4. Graphs of signal intensity were obtained through band densitometry and referred to GAPDH and control levels. Data are representative of three independent experiments and expressed as mean ± SD. P > 0.05 indicates non-significance; ***P < 0.001; **P < 0.01; *P < 0.05.

**Figure 4:** Effect of Eupafolin on PI3K/AKT, MAPKs and NF-κB signaling in breast cancer cells. (**A**,**B**) Eupafolin treatment leads to decreased phosphorylation of PI3K/AKT, Erk1/2, p38, and NF-κB/p65 by western blotting. Full-length images are presented in Supplementary Figs. 5 and 6. Graphs of signal intensity were obtained through band densitometry and referred to GAPDH and control levels. Data is representative of three independent experiments and expressed as mean ± SD. P > 0.05 indicates non-significance; ***P < 0.001; **P < 0.01; *P < 0.05.

### Anti-angiogenic activity of Eupafolin

Angiogenesis is very important in the development of cancer^14^. Thus, we tested the effect of Eupafolin on angiogenesis. First, results from the CCK8 experiment and cell colony formation assay demonstrated that the inhibitory effect of Eupafolin on HUVECs cell viability was dose-dependent (Fig. 5A,B). Second, results demonstrated that Eupafolin treatment was able to increase the apoptotic rate of HUVECs (Fig. 5C). Transwell assays were able to detect the migration and invasion ability of cells^15^. The migration and invasion ability of HUVECs decreased as the dose of Eupafolin increased (Fig. 5D). Endothelial cells have the ability to develop tubular structures and can therefore be used as screening drugs for anti-angiogenic activity^16^, Eupafolin treatment prevented the tube formation ability of HUVECs (Fig. 5E). Therefore, these results indicate that Eupafolin may be able to inhibit the formation of blood vessels.

**Figure 5:** Anti-angiogenic activity of Eupafolin. (**A**,**B**) Human umbilical vein endothelial cells (HUVECs) were treated with Eupafolin at concentrations of 0, 25, 50 and 100 μM for 24, 48, and 72 h, respectively. Cell viability was evaluated by the CCK-8 assay and cell colony formation assay. (**C**) HUVECs were treated with Eupafolin at concentrations of 0, 50, and 100 μM for 24 h, and then subjected to apoptotic analysis by flow cytometry (lower panel). (**D**) HUVECs treated with Eupafolin at concentrations of 0, 10, and 20 mg/ml were subjected to the migration and invasion assay and observed at 24 h, respectively. (**E**) HUVECs treated with Eupafolin at concentrations of 0, 50, and 100 μM for 6 h were subjected to the tube formation assay. Data is representative of three independent experiments and expressed as mean ± SD. P > 0.05 indicates non-significance; ***P < 0.001; **P < 0.01; *P < 0.05.

### Cavolin-1 involves in the regulation of Eupafolin

Firstly, we found that Eupafolin treatment led to a decrease in mRNA and protein expression of Cavolin-1 (Cav-1) in breast cancer cells (Fig. 6A,B). Cav-1 has recently been shown to mediate tumorigenesis and progression^17^. Thus, we set out to determine whether Cav-1 is involved in anti-proliferation effects of Eupafolin on breast cancer cells. Hence, we knocked down the expression of Cav-1 by transfecting Cav-1 siRNA into breast cancer cells (Fig. 6C). Among the two cell types, CCK8 results demonstrated showed that Cav-1 siRNA is able to inhibit the viability of MCF-7 cells when introduced into Cav-1 siRNA for 72 h. Furthermore, Cav-1 siRNA is able to reverse the cell viability inhibitory effect caused by Eupafolin (Fig. 6D,E).

**Figure 6:** Reduced Cav-1 is partially responsible for inhibition of proliferation of human breast cancer cells exposed to Eupafolin. (**A**,**B**) Total RNA and protein extracted from MDA-MB-231and MCF-7 cells treated with or without Eupafolin 50, and 100 μM for 24 h were used for quantitative real-time PCR and Western blot. Full-length images are presented in Supplementary Fig. 7. (**C**) MDA-MB-231and MCF-7 cells were transfected with Cav-1 siRNAs for 48 h and then subjected to Western Blot for evaluation of Cav-1 expression. Full-length images are presented in Supplementary Fig. 8. (**D**,**E**) MDA-MB-231and MCF-7 cells transfected with Cav-1 siRNAs or negative control siRNAs were treated with or without Eupafolin. Graphs of signal intensity were obtained through band densitometry and referred to GAPDH and control levels. Data are representative of three independent experiments and expressed as the mean ± SD. P > 0.05 indicates non-significance; ***P < 0.001; **P < 0.01; *P < 0.05.

### Eupafolin inhibited tumor growth in vivo

We established a xenograft tumor model using the human breast cancer MCF-7 cell line. When the tumor reached a volume of 50 mm^3^, the mice were administered an intraperitoneal injection of Eupafolin at a daily dose of 50 mg/kg. After 14 days, we found that Eupafolin significantly reduced the tumor volume, but had almost no effect on the weight of nude mice (Fig. 7A,B). Moreover, Eupafolin demonstrated no obvious toxicity on the major organs of nude mice. These results indicate that Eupafolin is able to effectively inhibit the progression of breast cancer in vivo.

**Figure 7:** Eupafolin inhibited the oncogenic capability of MCF-7 cells in nude mouse xenografts. (**A**) Nude mice bearing MCF-7 tumor xenografts were treated with Eupafolin (50 mg/kg, once daily, intraperitoneal injection). (**B**) Body weight of nude mice. (**C**) Schematic diagram of the potential molecular mechanism of Eupafolin-induced anticancer effect. The interaction between Eupafolin and PI3K/AKT, MAPKs and NF-κB is demonstrated. Data are representative of three independent experiments and expressed as mean ± SD. P > 0.05 indicates non-significance; ***P < 0.001; **P < 0.01; *P < 0.05.

## Discussion

Eupafolin is a natural compound that is extracted from plants. Previous studies have reported that Eupafolin has both anti-inflammatory and anti-tumor effects^18^. However, the role of Eupafolin in breast cancer, and its possible underlying mechanism of action, is not yet clear. Our results demonstrated that Eupafolin treatment had a significant inhibitory effect on breast cancer cell growth and development. By reducing the expression of Bcl-2 and increasing expression of Bax, cleaved caspase-3, LC3B-II and Beclin-1, Eupafolin was able to induce apoptosis, autophagy and S phase arrest. Moreover, Eupafolin-induced autophagy and apoptosis of breast cancer cells can be increased by RA and inhibited by 3-MA. Additionally, Cav-1 at least partially mediates Eupafolin-promoted inhibition of human breast cancer cell proliferation. In vivo, Eupafolin treatment significantly reduces tumor growth. Hence, the data indicates that Eupafolin inhibits growth and development of breast cancer cells by modulating the PI3K/Akt, MAPKs and NF-κB signaling pathway, which can be partially mediated by downregulated Cav-1 expression.

The cell cycle disorder that causes abnormal cell proliferation is one of the main mechanisms associated with tumorigenesis, and consisting of four distinct sequential phases. The S-phase within the DNA synthesis phase is the time it takes for DNA replication^19^. Therefore, it is important to cell cycle. Herein, we found that Eupafolin markedly induces cell-cycle arrest in S phase. Many traditional Chinese medicine monomers are also able to inhibit proliferation of cancer cells by blocking cells in the S-phase, such as Quercetin^20^, Baicalein^21^ and Daidzein^22^. Moreover, the expressions of Cyclins, and CDKs are related to cell cycle^23^. For example, The down-regulation of CDK2, CDK4 and Cyclin B1 can be inhibited by the development of breast cancer^24^.

Apoptosis plays a vital role in cell survival^25^. Caspase-3 is the most important terminal splicing enzyme in apoptosis and has an important part in the mechanism leading to cell death^26^. In addition, previous studies have shown that the Bcl-2 family inhibits mitochondrial-induced apoptosis^27^. Moreover, Eupafolin is able to promote apoptosis of cervical and renal cancer cells^28^. In this study, we found that Eupafolin has the same effect in breast cancer cells.

In order to further understand the anti-cancer mechanisms of Eupafolin in breast cancer cells, we determined protein levels in the PI3K/AKT pathway that were involved in tumor cell growth, differentiation, and apoptosis^29^. Herein, results from Western blot analysis demonstrated that Eupafolin significantly blocked phosphorylation of the PI3K/AKT signaling pathway. Moreover, the activity of p38 signaling can induce autophagy^30^. Herein, Eupafolin promotes the role of p38. ERK and p38 are members of the MAPK family. According to reports, activation of MAPK is able to inhibit the proliferation of cancer cells^31^. These results demonstrated that Eupafolin treatment activated MAPK signaling pathway in breast cancer cells. Therefore, down-regulation of MAPK is partially related to induction of apoptosis in breast cancer cells by Eupafolin treatment.

The migration and invasion of tumor cells is one of the main problems in the treatment process^32^. In our study, we found that Eupafolin is able to inhibit the metastatic ability of breast cancer cells. Previous studies have shown that angiogenesis can promote tumor growth and metastasis. Therefore, inhibition of tumor angiogenesis can be a good treatment for cancer. The anti-angiogenesis ability of a drug can be effectively evaluated by detecting the activity on endothelial cells^33^. In addition, we tested cellular proliferation, apoptosis, migration, invasion, colony formation and tube formation assay of Eupafolin in HUVECs^34^. Caveolin (Cav-1) is a subdomain rich in the plasma membrane, and its expression is out of control in cancer cells^35^. Cav-1 is thought to be involved in the regulation of several biological processes in both normal tissues and cancer. According to reports, Cav-1 can function to promote and suppress tumors, according to the type of cancer cells^36^. Our study demonstrated that Eupafolin inhibited Cav-1 expression in breast cancer cells. Moreover, down-regulation of Cav-1 contributes to the inhibition of proliferation of MCF-7 cells that were exposed to Eupafolin, and Cav-1 siRNA is able to reverse the cell viability inhibitory effect caused by Eupafolin. Therefore, the anti-breast cancer activity of Eupafolin is partially mediated by Cav-1.

Collectively, this study suggests that Eupafolin significantly inhibits breast cancer cell growth and development, and promotes autophagy via the PI3K/AKT, MAPKs and NF-κB signaling pathways. Mechanistically, Eupafolin exerts anti-breast cancer activity partially through down regulation of Cav-1. Moreover, Eupafolin has beneficial anti-cancer effects within the body. The interaction between Eupafolin and PI3K/AKT, MAPKs and NF-κB is shown in Fig. 7C. Therefore, our results provide a theoretical basis for use of Eupafolin in clinical trials.

## Supplementary Information

Supplementary Figures.

## Data Availability

The datasets used and/or analyzed during the current study are available from the corresponding author on reasonable request.

## References

[1] Watkins EJ (2019). Overview of breast cancer. JAAPA.

[2] Nanda R, Chow LQ, Dees EC, Berger R, Gupta S, Geva R, Pusztai L, Pathiraja K, Aktan G, Cheng JD, Karantza V, Buisseret L (2016). Pembrolizumab in patients with advanced triple-negative breast cancer: Phase Ib KEYNOTE-012 study. J. Clin. Oncol..

[3] Chung KS, Choi JH, Back NI, Choi MS, Kang EK, Chung HG, Jeong TS, Lee KT (2010). Eupafolin, a flavonoid isolated from Artemisia princeps, induced apoptosis in human cervical adenocarcinoma HeLa cells. Mol. Nutr. Food Res..

[4] Folkman J (1972). Anti-angiogenesis: New concept for therapy of solid tumors. Ann. Surg..

[5] Hamurcu Z, Delibasi N, Gecene S, Sener EF, Donmez-Altuntas H, Ozkul Y, Canatan H, Ozpolat B (2018). Targeting LC3 and Beclin-1 autophagy genes suppresses proliferation, survival, migration and invasion by inhibition of Cyclin-D1 and uPAR/Integrin beta1/ Src signaling in triple negative breast cancer cells. J. Cancer Res. Clin. Oncol..

[6] Zhang H, Zhu Y, Sun X, He X, Wang M, Wang Z, Wang Q, Zhu R, Wang S (2016). Curcumin-loaded layered double hydroxide nanoparticles-induced autophagy for reducing glioma cell migration and invasion. J. Biomed. Nanotechnol..

[7] Wu Z, Zhu Q, Yin Y, Kang D, Cao R, Tian Q, Zhang Y, Lu S, Liu P (2018). Traditional Chinese Medicine CFF-1 induced cell growth inhibition, autophagy, and apoptosis via inhibiting EGFR-related pathways in prostate cancer. Cancer Med..

[8] Wu M, Lao Y, Xu N, Wang X, Tan H, Fu W, Lin Z, Xu H (2015). Guttiferone K induces autophagy and sensitizes cancer cells to nutrient stress-induced cell death. Phytomedicine.

[9] Wang G, Wang T, Zhang Y, Li F, Yu B, Kou J (2019). Schizandrin protects against OGD/R-induced neuronal injury by suppressing autophagy: Involvement of the AMPK/mTOR pathway. Molecules.

[10] Yang PW, Lu ZY, Pan Q, Chen TT, Feng XJ, Wang SM, Pan YC, Zhu MH, Zhang SH (2019). MicroRNA-6809-5p mediates luteolin-induced anticancer effects against hepatoma by targeting flotillin 1. Phytomedicine.

[11] Fresno Vara JA, Casado E, de Castro J, Cejas P, Belda-Iniesta C, Gonzalez-Baron M (2004). PI3K/Akt signalling pathway and cancer. Cancer Treat. Rev..

[12] Livak KJ, Schmittgen TD (2001). Analysis of relative gene expression data using real-time quantitative PCR and the 2(-Delta Delta C(T)) Method. Methods.

[13] Dong H, Diao H, Zhao Y, Xu H, Pei S, Gao J, Wang J, Hussain T, Zhao D, Zhou X, Lin D (2019). Overexpression of matrix metalloproteinase-9 in breast cancer cell lines remarkably increases the cell malignancy largely via activation of transforming growth factor beta/SMAD signalling. Cell Prolif..

[14] Li Y, Zhou D, Ren Y, Zhang Z, Guo X, Ma M, Xue Z, Lv J, Liu H, Xi Q, Jia L, Zhang L, Liu Y, Zhang Q, Yan J, Da Y, Gao F, Yue J, Yao Z, Zhang R (2019). Mir223 restrains autophagy and promotes CNS inflammation by targeting ATG16L1. Autophagy.

[15] Tewari KS, Sill MW, Long HJ, Penson RT, Huang H, Ramondetta LM, Landrum LM, Oaknin A, Reid TJ, Leitao MM, Michael HE, Monk BJ (2014). Improved survival with bevacizumab in advanced cervical cancer. N. Engl. J. Med..

[16] Tripathy J, Tripathy A, Thangaraju M, Suar M, Elangovan S (2018). alpha-Lipoic acid inhibits the migration and invasion of breast cancer cells through inhibition of TGFbeta signaling. Life Sci..

[17] Chen X, Zhao Y, Yang A, Tian Y, Pang D, Sun J, Tang L, Huang H, Wang Y, Zhao Y, Tu P, Hu Z, Li J (2020). Chinese Dragon's blood EtOAc extract inhibits liver cancer growth through downregulation of Smad3. Front. Pharmacol..

[18] Wang S, Wang N, Zheng Y, Zhang J, Zhang F, Wang Z (2017). Caveolin-1: An oxidative stress-related target for cancer prevention. Oxid. Med. Cell Longev..

[19] Dumont NA, Wang YX, von Maltzahn J, Pasut A, Bentzinger CF, Brun CE, Rudnicki MA (2015). Dystrophin expression in muscle stem cells regulates their polarity and asymmetric division. Nat. Med..

[20] Chou CC, Yang JS, Lu HF, Ip SW, Lo C, Wu CC, Lin JP, Tang NY, Chung JG, Chou MJ, Teng YH, Chen DR (2010). Quercetin-mediated cell cycle arrest and apoptosis involving activation of a caspase cascade through the mitochondrial pathway in human breast cancer MCF-7 cells. Arch. Pharm. Res..

[21] Gao J, Morgan WA, Sanchez-Medina A, Corcoran O (2011). The ethanol extract of *Scutellaria baicalensis* and the active compounds induce cell cycle arrest and apoptosis including upregulation of p53 and Bax in human lung cancer cells. Toxicol. Appl. Pharmacol..

[22] Wang HZ, Zhang Y, Xie LP, Yu XY, Zhang RQ (2002). Effects of genistein and daidzein on the cell growth, cell cycle, and differentiation of human and murine melanoma cells(1). J. Nutr. Biochem..

[23] Spring LM, Wander SA, Zangardi M, Bardia A (2019). CDK 4/6 inhibitors in breast cancer: Current controversies and future directions. Curr. Oncol. Rep..

[24] Sheng YN, Luo YH, Liu SB, Xu WT, Zhang Y, Zhang T, Xue H, Zuo WB, Li YN, Wang CY, Jin CH (2020). Zeaxanthin induces apoptosis via ROS-regulated MAPK and akt signaling pathway in human gastric cancer cells. Onco Targets Ther..

[25] Xu F, Li Q, Wang Z, Cao X (2019). Sinomenine inhibits proliferation, migration, invasion and promotes apoptosis of prostate cancer cells by regulation of miR-23a. Biomed. Pharmacother..

[26] Shalini S, Dorstyn L, Dawar S, Kumar S (2015). Old, new and emerging functions of caspases. Cell Death Differ..

[27] Siddiqui WA, Ahad A, Ahsan H (2015). The mystery of BCL2 family: Bcl-2 proteins and apoptosis: An update. Arch. Toxicol..

[28] Han MA, Min KJ, Woo SM, Seo BR, Kwon TK (2016). Eupafolin enhances TRAIL-mediated apoptosis through cathepsin S-induced down-regulation of Mcl-1 expression and AMPK-mediated Bim up-regulation in renal carcinoma Caki cells. Oncotarget.

[29] Nan Y, Guo H, Guo L, Wang L, Ren B, Yu K, Huang Q, Zhong Y (2018). MiRNA-451 inhibits glioma cell proliferation and invasion through the mTOR/HIF-1alpha/VEGF signaling pathway by targeting CAB39. Hum. Gene Ther. Clin. Dev..

[30] Kim KY, Park KI, Kim SH, Yu SN, Park SG, Kim YW, Seo YK, Ma JY, Ahn SC (2017). Inhibition of autophagy promotes salinomycin-induced apoptosis via reactive oxygen species-mediated PI3K/AKT/mTOR and ERK/p38 MAPK-dependent signaling in human prostate cancer cells. Int. J. Mol. Sci..

[31] Fang JY, Richardson BC (2005). The MAPK signalling pathways and colorectal cancer. Lancet Oncol..

[32] Ren S, Liu J, Feng Y, Li Z, He L, Li L, Cao X, Wang Z, Zhang Y (2019). Knockdown of circDENND4C inhibits glycolysis, migration and invasion by up-regulating miR-200b/c in breast cancer under hypoxia. J. Exp. Clin. Cancer Res..

[33] Jaszai J, Schmidt MHH (2019). Trends and challenges in tumor anti-angiogenic therapies. Cells.

[34] Bejar MT, Ferrer-Lorente R, Pena E, Badimon L (2016). Inhibition of Notch rescues the angiogenic potential impaired by cardiovascular risk factors in epicardial adipose stem cells. FASEB J..

[35] Liang W, Hao Z, Han JL, Zhu DJ, Jin ZF, Xie WL (2014). CAV-1 contributes to bladder cancer progression by inducing epithelial-to-mesenchymal transition. Urol. Oncol..

[36] Vykoukal J, Fahrmann JF, Gregg JR, Tang Z, Basourakos S, Irajizad E, Park S, Yang G, Creighton CJ, Fleury A, Mayo J, Paulucci-Holthauzen A, Dennison JB, Murage E, Peterson CB, Davis JW, Kim J, Hanash S, Thompson TC (2020). Caveolin-1-mediated sphingolipid oncometabolism underlies a metabolic vulnerability of prostate cancer. Nat. Commun..

